RETRACTED

# Effects of Self-Made Prescription Compound Rhodiola on the Ultrastructure of Podocytes in Rats with Type 2 Diabetic Nephropathy

**DOI:** 10.1155/2022/3417557

**Published:** 2022-06-22

**Authors:** Shaojing Yuan, Jie Liu, Zhenhua Sun, Lihua Meng, Jiying Zhu, Min Wang, Jie Su

**Affiliations:** ^1^The University of Shandong of Traditional Chinese Medicine, Jinan, Shandong 250355, China; ^2^Department of Community Health Management, The Second Affiliated Hospital of Shandong University of Traditional Chinese Medicine, Jinan, Shandong 250355, China; ^3^Department of Nephropathy and Oncology, Three Departments of Traditional Chinese Medicine Hospital of Mengyin County, Linyi, Shandong 276200, China; ^4^Department of Cadre Health Care, The Second Affiliated Hospital of Shandong University of Traditional Chinese Medicine, Jinan, Shandong 250001, China; ^5^The Second Affiliated Hospital of Shandong University of Traditional Chinese Medicine, Jinan, Shandong 250001, China

## Abstract

**Background:**

We attempt to discuss the function of self-made prescription compound Rhodiola rosea on the kidneys of rats with type 2 diabetic nephropathy (DN), through studying the effects of self-made rescription compound Rhodiola rosea on the ultrastructure of podocytes in rats with DN.

**Methods:**

DN rat model was established by streptozotocin. The successfully modeled rats were divided into 4 groups, DN group, compound Rhodiola low-dose group, medium-dose group, and high-dose group. Compound Rhodiola low-dose group, medium-dose group, and high-dose group were administered for 8 weeks, and the DN group and the blank control group were administered with normal saline. The podocyte count, podocyte width, podocyte fusion rate, and average thickness of glomerular basement membrane were compared in each group, and the ultrastructural changes in podocytes were observed by transmission electron microscope.

**Results:**

Compared with the normal control group, the number of podocytes in the DN group remarkably reduced, but the width level of podocyte, the fusion rate of podocyte, and the average thickness of basilar membrane remarkably increased (*P* < 0.05). Compared with the DN group, the number of podocytes in the high-, medium-, and low-dose groups increased remarkably, but the width level of podocyte, the fusion rate of podocyte, and the average thickness of basilar membrane decreased remarkably (*P* < 0.05). Compared with the low-dose group, the number of podocytes in the high-dose group and the medium-dose group increased remarkably, but the width of podocyte, the fusion rate of podocyte, as well as the average thickness of basilar membrane remarkably reduced (*P* < 0.05). Various indicators of high- and medium-dose groups had no statistical difference (*P* > 0.05).

RETRACTED

**Conclusions:**

Self-made prescription compound Rhodiola rosea can promote the recovery of podocyte in DN rat and protect their kidney.

## 1. Introduction

As technology advances, the global economy is in a stage of rapid development. The living standards of human beings are constantly improving, and the lifestyles are constantly changing. The threat of chronic diseases to human health is increasing day by day, and the incidence of diabetes mellitus (DM) is increasing rapidly in countries around the world. According to the International Diabetes Federation statistics, the number of people with DM in the world was about 366 million in 2011, and the number of people with DM is estimated to increase to 552 million by 2030 [1]. China has witnessed one of the most dramatic rises in diabetes prevalence anywhere in the world, with 23.8 million DM patients, and it is expected to exceed 42.3 million in 2030 [2, 3]. Diabetic nephropathy (DN) is a common and frequent clinical complication of DM. Approximately 30% to 40% of individuals with diabetes mellitus develop DN. According to statistics, all-cause mortality in individuals with DN is approximately 30 times higher than that in diabetic patients without nephropathy [5]. DN has become the second leading cause of end-stage renal disease and one of the leading causes of death in diabetic patients [6]. The changes in the ultrastructure of renal podocytes and the changes in the expression of related molecules play an important role in diabetic nephropathy development [7]. Rhodiola rosea has anti-inflammatory, anticancer, antioxidation, and other pharmacological effects. However, whether Rhodiola rosea plays a beneficial role in diabetic nephropathy remains unclear [8]. This study aimed to discuss the effects of self-made prescription compound Rhodiola rosea on the kidney podocytes and their ultrastructure of DN rats through animal experiments and also their effects on the kidneys of DN rats.

## 2. Research Content and Methods

### 2.1. Materials and Reagents

#### 2.1.1. Experimental Animals

58-week-old SPF male Wistar rats (weight 200–220 g) were purchased from the Experimental Animal Center of Shandong University.

#### 2.1.2. Experimental Reagents

Streptozotocin (STZ) and its solution preparation materials (citric acid, sodium citrate, distilled water) are produced by American Sigma Company. The urine microalbumin (mALB) assay kit is produced by Orion Diagnostica Oy, Finland, and purchased from Beijing Northern Institute of Biotechnology. The fixing reagent (3% glutaraldehyde, 1% osmic acid), dehydrating agent (50% ethanol, 70% ethanol, 90% ethanol, 90% acetone, 90% ethanol: 90% acetone = 1 : 1 mixture), embedding agent (Epon 812 epoxy resin embedding agent), and electronic staining agent (uranyl acetate, lead citrate) were prepared by the electron microscope room of Medical College of Shandong University. Light microscope staining solution (0.5% toluidine blue) is provided by the electron microscope room of Medical College of Shandong University.

RETRACTED

#### 2.1.3. Experimental Instruments

The biochemical analyzer was provided by the Second Affiliated Hospital of Shandong University of Traditional Chinese Medicine, and the model is Hitachi 7600 Series, the automatic biochemical analyzer (made in Japan). The transmission electron microscope was provided by the electron microscope room of Medical College of Shandong University, model: JME-d-1200EX (made in Japan), resolution: 0.1–10 nm, and acceleration voltage: 60–100 kV. The ultrathin slicer was provided by the electron microscope room of Medical College of Shandong University, and the model is Ultracut E, Cambridge, UK.

#### 2.1.4. Experimental Prescription

Self-made prescription compound Rhodiola was purchased from the Affiliated Hospital of Shandong University of Traditional Chinese Medicine. Compound Rhodiola rosea is a powder made by drying Rhodiola rosea dry root and astragalus root as the main raw materials, soluble starch, corn starch, ethanol, and other auxiliary materials at 50°C.

#### 2.1.5. High-Glucose and High-Lipid Fodder Formula

High-glucose and high-lipid fodder formula consists of 3% egg yolk, 18% lard, 20% sucrose, and 59% basic feed, processed by Shandong Lukang Pharmaceutical Co., Ltd. (SCXK Lu 20080002).

### 2.2. Experimental Steps

#### 2.2.1. Feeding Period

Fifty rats were divided into the normal control group (*n* = 5) and the model experimental group (*n* = 45). The normal control group was fed with normal diet for 8 weeks, and the model experimental group was fed with high-glucose and high-lipid fodder for 8 weeks. All rats were housed at 55% ± 5% humidity and constant room temperature (22–24°C), under a controlled light cycle. All animals were free to drink water. The animal procedures were in accordance with the Experimental Animal Center of Shandong University.

#### 2.2.2. Construction of Diabetic Nephropathy Rat Model

Model experimental group rats were fed for 8 weeks and had no eating and no drinking for 16 hours. After that, STZ (30 mg/kg) was rapidly injected in the left abdominal cavity. Normal control group was injected with the same volume of sodium citrate buffer. After 1 week of fasting for 12 hours, blood is fetched from rat tail vein to measure fasting blood glucose (FBG) and fasting insulin (FINS) and the insulin resistance index is calculated (HOMA-IR) (formula: HOMA-IR = (FBG (mmol/l)*∗*FINS (mu/l))/22.5). Criteria for successful modeling of diabetic nephropathy are as follows: FBG ≥ 7.0 mmL/L, HOMA-IR higher than the normal control group, and 12 h urinary microalbumin ≥30 mg/L. In this experiment, 43 rat DN models were successfully established.

RETRACTED

#### 2.2.3. Grouping and Treatment

Forty-three successful modeling DN rats were randomly divided into 4 groups: DN group (*n* = 10), compound Rhodiola low-dose (*n* = 11), medium-dose (*n* = 11), and high-dose (*n* = 11) groups. The normal control group and the DN group are perfused with 2 ml of normal saline every day. Compound Rhodiola of 3, 6, and 12 g/(kg·D) was dissolved in 2 ml normal saline and stirred evenly, and then, the rats in the low-, medium-, and high-dose groups were given intragastric administration for 4 weeks, respectively. During the whole experimental process, all groups were not given insulin and hypoglycemic drugs. After 4 weeks, only 35 rats were alive, DN group (*n* = 9), compound Rhodiola low-dose group (*n* = 9), medium-dose group (*n* = 9), and high-dose group (*n* = 8).

#### 2.2.4. Collection of Kidney Specimens from Rats

After 4 weeks of treatment, the rats were anesthetized, and the kidneys of the rats in each group were removed. Kidneys were isolated, fixed within 1 min, and then quickly placed into a 9% saline rinse bottle to remove blood and mucus, and absorbent paper was used to absorb excess water. The renal cortex (the outermost layer of the upper pole of the kidney) was placed on ice, and the renal cortex was rinsed with 0.1% phosphate-buffered saline (PB). The tissue was cut into small pieces of about 1 mm × 1 mm × 1 mm, fixed in 3% glutaraldehyde fixative solution at low temperature (0–4°C) for 2 hours, and post-fixed with 1% osmic acid for 1 hour, and the tissues were dehydrated, infiltrated, embedded, aggregated, sectioned, and stained.

### 2.3. Observation Indicators

In this experiment, we observed the rat kidney tissue by transmission electron microscope, and the observation indicators were average thickness of podocyte fusion rate and glomerular basement membrane (GBM), average width of podocyte (FPW), and podocyte counting. Under the electron microscope ×5000 times, 3 glomeruli of each case were observed, and 10 visual fields randomly from each glomerulus are obtained, and the number of podocytes is calculated. Under the electron microscope ×10000 times, 20 podocytes were randomly selected from each case, the distance between the membranes on both sides of the podocyte between the two-hole membranes was measured, and the average value was taken. Under the electron microscope ×10000 times, with 2 *μ*m as the unit, 20 measurement units were randomly selected for each case, the total length of basement membrane *Y* = 40 *μ*m, and then the total length of podocyte fusion on the basement membrane is measured, *X* is set, and finally *X*/*Y* is adopted, and we could obtain the fusion rate. Under the electron microscope ×10000 times, with 1 *μ*m as the unit, 20 measurement units were randomly selected for each case, and 3 points were randomly found in each unit to measure the thickness of basement membrane at each point, then all the thicknesses are added and set as *X*, the number of measured points was set as *Y*, finally *X*/*Y* is adopted, and then we obtained the average thickness of each group of basement membranes.

RETRACTED

### 2.4. Data Statistics

We analyzed all data by SPSS 18 0 software. We expressed all data obtained by mean ± standard deviation and compared the differences between both groups by *t*-test and the differences among multiple groups by analysis of variance. When *P* < 0.05, it possessed statistical significance.

## 3. Results

### 3.1. Comparison of Podocyte Count, the Width of Podocyte, the Fusion Rate of Podocyte, and the Thickness of GBM in Each Group of Rats

The results showed that in contrast to the normal control group, the number of podocytes in the DN group remarkably decreased, but the width level of podocyte, the fusion rate of podocyte, and the average thickness of basement membrane remarkably increased, and it possessed statistical significance (*P* < 0.05) (Tables 1 and 2).

Compared with the DN group, the number of podocytes in the high-, medium-, and low-dose groups increased remarkably, but the width of podocyte, the fusion rate of podocyte, and the average thickness of GBM remarkably decreased, with statistical significance (*P* < 0.05). Comparison among the high-, medium-, and low-dose groups: compared with the low-dose group, the number of podocytes in the high- and medium-dose groups was significantly increased, and the width of podocyte, the fusion rate of podocyte, and the average thickness of GBM were significantly decreased, and it possessed statistical significance (*P* < 0.05). Various indexes of the high- and medium-dose groups had no statistical difference (*P* > 0.05).

### 3.2. Comparison of Ultrastructural Images of Renal Podocytes

The results of the normal control group showed that the glomerular basement membrane was clear, the thickness was uniform, and there was no obvious thickening. The podocyte was clear and neatly arranged, with no fusion or reduction in the podocyte, and the width of podocyte was normal (Figure 1). On the contrary, the glomerular basement membrane of rats in the DN group remarkably thickened, and a double-track phenomenon appeared. The basement membrane had large dense deposits with different thicknesses, and the width of podocyte is irregularly arranged. The podocyte was obviously fused, and inflammatory cells appeared (Figure 2). In the low-dose group, the thickening of GBM, the width of podocyte, flattening, reduction, and irregular arrangement of rats had not remarkably reduced (Figure 3). In the medium-dose group, GBM was thickened, the width of podocyte was irregularly arranged, and the fusion rate of podocyte and other phenomena were significantly alleviated (Figure 4). The glomerular basement membrane of the rats in the high-dose group was thickened and irregularly arranged, and the phenomenon of flattening, fusion, and reduction in the podocyte was also significantly improved, and it had no obvious difference compared with the medium-dose group (Figure 5).

RETRACTED

Compound Rhodiola rosea can increase the number of podocytes in type 2 diabetic nephropathy rats, reduce the width of podocyte, the fusion rate of podocyte, and the average thickness of GBM. The medium- and high-dose groups have a better therapeutic effect than the low-dose group, indicating that compound Rhodiola rosea can repair renal podocytes in DN rats.

## 4. Discussion

At present, the etiology and mechanism of DN are not completely clear, and its occurrence and development are the result of the combined effect of multiple factors. It is now believed that there is a certain correlation with many factors such as genetics, hemodynamic disorders, lipid metabolism disorders, stress response, and hypertension. Various comprehensive factors eventually lead to DN. Podocytes are the largest cells in the glomerulus, which are attached to the outside of the GBM, showing a multi-protrusion shape. The fissure between adjacent podocytes is covered by a thin film called the slit membrane. Podocytes and slit membranes are one of the important components of the glomerular filtration membrane. Studies have shown that podocyte injury plays a key role in the pathogenesis of DN [9, 10]. The number and density of podocytes in the early stage of DN have begun to decrease and worsen with the aggravation of the disease [11]. The density and total number of podocytes are reduced by apoptosis and shedding due to injury, and the residual podocyte widens and fuses, resulting in compensatory hypertrophy, leading to glomerular sclerosis and destruction of the glomerular filtration barrier [12]. Once podocytes are damaged and fall off, they lack the ability to regenerate [9]. Therefore, podocyte repair plays a crucial role in DN treatment.

RETRACTED

Rhodiola is a very important natural wild plant in Tibetan medicine in my country, with unique biological effects. Modern research has shown that Rhodiola rosea not only has the functions of clearing the lungs and relieving cough, invigorating Qi, and promoting blood circulation, but also anti-hypoxia, antiaging, and antitumor [13–15]. In this experiment, we further studied its effect on renal podocytes and their ultrastructure in DN rats. The results showed that compared with the normal control group, the number of podocytes in the DN group was significantly less, and the width level of podocyte, the fusion rate of podocyte, and the average thickness of basement membrane were significantly higher, which was supported by the ultrastructure of podocyte. Based on the above observations, the rat model was successfully replicated. Compared with the model of control group, the number of podocytes in the high-, medium-, and low-dose groups increased significantly, and the width of podocyte, the fusion rate of podocyte, and the average thickness of GBM decreased significantly, which was supported by the ultrastructure of podocytes, indicating that the podocytes of DN rats treated with self-made compound Rhodiola gradually repaired. Compared with the low-dose group, the high- and medium-dose groups had significantly more podocytes, and the width of podocyte, the fusion rate of podocyte, and average thickness of GBM were significantly lower, which was corroborated with the podocyte ultrastructure. The experiment proved that the effect of high- and medium-dose groups in promoting the ultrastructure of renal podocytes of DN rats to return to normal was better than that of the low-dose group. The self-made prescription compound Rhodiola rosea is mainly composed of Rhodiola rosea, Radix Astragali, and other traditional Chinese medicines for supplementing Qi and activating blood circulation. In this study, compound Rhodiola rosea was used to treat DN from the perspective of nourishing Qi and activating blood circulation. Rhodiola rosea extract can significantly improve the thickening of rat GBM and protect the kidneys of DM rats. Rhodiola rosea alleviated high-glucose-induced oxidative stress and extracellular matrix accumulation in rat glomerular mesangial cells by the TXNIP-NLRP3 inflammasome pathway [16]. Radix Astragali can improve podocyte adhesion function, reduce blood glucose and urinary protein, and further slow down the progression of DN [17]. Rhodiola rosea extract may have a protective effect on early nephropathy in diabetic rats [18].

## 5. Conclusion

To sum up, the changes in podocyte ultrastructure in normal rats, DN rats, and DN rats treated with Rhodiola rosea were observed under the electron microscope in this subject. From the pathological point of view, we explored the effect of compound Rhodiola rosea in repairing renal ultrastructure to protect the kidneys and explained the mechanism of the self-made prescription compound Rhodiola in the effective treatment of DN. It has important guiding significance for the clinical treatment of diabetic nephropathy and lays a certain experimental foundation for the development of Chinese medicine in treating DN. In addition, studying the target of compound Rhodiola in podocytes from molecular biology will also become the next research direction of our research group.

RETRACTED

## Figures and Tables

**Figure 1:** Normal control group. (a) Basement membrane is even and clear, podocyte in order and without fusion or decreasing. (b) Junction of three vascular cavities, podocyte without fusion or decreasing. (c) No basement membrane thickening.

**Figure 2:** DN group. (a) Double-rail phenomenon appears in basement membrane, quantities of podocyte reduced and fused. (b) Podocyte flatted, fused, decreased, podocyte width enlarged, inflammatory cells of mesangial region appeared. (c) Basement membrane had plenty of dense deposits and it was vague and unclear, podocyte flatted, decreased, podocyte width enlarged.

**Figure 3:** Low-dose group. (a) Podocyte fused obviously, podocyte flatted, decreased, podocyte width enlarged. (b) Flaky dense deposits, basement membrane thickened obviously. (c) Podocyte fused, flatted, decreased, podocyte width enlarged.

**Figure 4:** Medium-dose group. (a) No obvious podocyte fused or flatted or decreased. (b) No basement membrane thickening, uniform thick and thin. (c) Uniform basement membrane, no podocyte decreasing.

**Figure 5:** High-dose group. (a) No basement membrane thickening, uniform, no podocyte fused or decreased. (b) Basement membrane thickness was uniform and clear, podocyte in order, no fusion. (c) No podocyte flatting, decreasing, basement membrane was clearly visible.

**Table 1:** Number of podocytes, the podocyte width, the podocyte fusion rate, and the average thickness of the GBM in the control group ($\bar{x}\pm s$).

Group	Number of podocytes	Width of the podocyte (um)	Fusion rate of the podocyte (%)	Average thickness of GBM (um)
Normal control group	10.30 ± 0.36	0.263 ± 0.022	3.10 ± 1.01	0.23 ± 0.02
DN group	1.20 ± 0.51	0.855 ± 0.034	65.80 ± 3.30	0.78 ± 0.11
*t*	43.730	43.860	54.500	14.760
*P*	<0.001	<0.001	<0.001	<0.001

DN: diabetic nephropathy; GBM: glomerular basement membrane.

**Table 2:** Number of podocytes, the width of the podocyte, the fusion rate of the podocyte, and the thickness of the GBM between the models in each group ($\bar{x}\pm s$).

Group	Number of podocytes	Width of the podocyte (um)	Fusion rate of the podocyte (%)	Average thickness of GBM (um)
DN group	1.2 ± 0.51	0.855 ± 0.034	65.8 ± 3.3	0.78 ± 0.11
Low-dose group	4.0 ± 0.34^*∗*^	0.391 ± 0.023^*∗*^	56.25 ± 7.8^*∗*^	0.51 ± 0.04^*∗*^
Medium-dose group	9.3 ± 0.27^*∗*Δ^	0.282 ± 0.021^*∗*Δ^	21.21 ± 5.4^*∗*Δ^	0.32 ± 0.12^*∗*Δ^
High-dose group	8.2 ± 0.24^*∗*Δ^	0.311 ± 0.032^*∗*Δ^	29.32 ± 1.8^*∗*Δ^	0.40 ± 0.22^*∗*Δ^

DN: diabetic nephropathy; GBM: glomerular basement membrane. ^*∗*^*P* < 0.05, compared with the DN group; ^Δ^*P* > 0.05, compared with the low-dose group.

RETRACTED

## Data Availability

The data can be obtained from the author upon reasonable request.
